The article "Similarities and Differences in Bone Mineral Density between Multiple Sites in the Same Individual: An Elderly Cadaveric Study" was published in 2022. Journal: Biomed Res Int.

# Similarities and Differences in Bone Mineral Density between Multiple Sites in the Same Individual: An Elderly Cadaveric Study

**DOI:** 10.1155/2022/6094663

**Published:** 2022-06-07

**Authors:** Keita Nishi, Daisuke Endo, Takashi Hasegawa, Takefumi Moriuchi, Keiko Ogami-Takamura, Kazunobu Saiki, Kiyohito Murai, Toshio Higashi, Toshiyuki Tsurumoto, Yoshitaka Manabe, Joichi Oyamada

**Affiliations:** ^1^Department of Oral Anatomy and Dental Anthropology, Graduate School of Biomedical Sciences, Nagasaki University, 1-7-1 Sakamoto, Nagasaki, Nagasaki 852-8588, Japan; ^2^Department of Macroscopic Anatomy, Graduate School of Biomedical Sciences, Nagasaki University, 1-12-4 Sakamoto, Nagasaki, Nagasaki 852-8523, Japan; ^3^Center of Cadaver Surgical Training, Nagasaki University School of Medicine, 1-12-4 Sakamoto, Nagasaki, Nagasaki 852-8523, Japan; ^4^Department of Health Science, Graduate School of Biomedical Sciences, Nagasaki University, 1-7-1 Sakamoto, Nagasaki, Nagasaki 852-8520, Japan; ^5^Department of Rehabilitation Sciences, Graduate School of Biomedical Sciences, Nagasaki University, 1-7-1 Sakamoto, Nagasaki, Nagasaki 852-8520, Japan

## Abstract

Bone mineral density (BMD) is known to vary based on various factors, and the degree of variation is site-specific. However, few studies have investigated the relationship between bone density at trabecular bone-rich and cortical bone-rich sites in the same individual. In this study, we attempted to measure BMD at multiple sites using whole-body computed tomography images taken immediately after death and to clarify the similarities and differences between skeletal sites. Additionally, we aimed to examine the factors that influence changes in BMD, such as the loading environment, bone microstructure, and the ossification process of each skeletal region. A 3D model containing BMD data of the skull, clavicle, lumbar vertebrae, and femur (neck and diaphysis) was created using computed tomography images taken immediately after the death of 60 individuals (28 men and 32 women, average age: 84.0 years) who consented to participate in the study before death. Arbitrary measurement sites were defined, and bone density was measured at each site. We found that the BMDs of all regions were negatively correlated with age, but this correlation was weaker in the skull than in other regions. The negative correlation was especially pronounced in areas with more trabecular bones in men and in areas with more cortical bones in women. Furthermore, these findings suggest that factors, such as the loading environment, bone microstructure, and the ossification process of the skeletal sites, affect the BMD. Furthermore, our results suggest that it is important to assess the BMD of cortical bone in older women.

The article "Similarities and Differences in Bone Mineral Density between Multiple Sites in the Same Individual: An Elderly Cadaveric Study" was published in 2022. Journal: Biomed Res Int.

## 1. Introduction

Osteoporosis is an age-related degenerative disease associated with fractures of the limb bones and spine, which significantly reduces the quality of life in elderly individuals [1–3]. Postmenopausal women have a high prevalence of osteoporosis, which contributes to the high incidence of fragility fractures among elderly women [4, 5]. Most research on osteoporosis has been focused on trabecular bone-rich sites, such as the vertebral column and femoral neck, which are the predominant sites for vulnerable fractures. However, in recent years, issues related to atypical femur fractures such as fatigue fractures in the subtrochanteric and proximal diaphysis areas have been reported in the elderly [6–8]. Fragility fractures caused due to decreased bone strength associated with increased porosity and decreased thickness of cortical bone have also been reported [9–12].

Bone mineral density (BMD) is one of the most important diagnostic criteria for osteoporosis and is measured by a variety of methods [13, 14]. Dual-energy X-ray absorptiometry is commonly used in clinical practice. However, this technique does not provide an adequate BMD based on the measurement site because it measures BMD per unit area, which is easily affected by body size and artifacts. In recent years, high-resolution peripheral quantitative computed tomography (HR-pQCT) has been frequently used for the analysis of cortical bone [15, 16]. However, HR-pQCT can only analyze peripheral bones, which makes it difficult to use for a wide range of sites. On the other hand, quantitative computed tomography (QCT) is a frequently used technique that can measure bone density per unit volume at any site of the body based on CT values (Hounsfield units) obtained from CT images [17]. Therefore, it is possible to obtain bone density data for several sites if whole-body CT images are available. However, due to radiation exposure issues, it is difficult to obtain the data unless absolutely necessary.

Therefore, this study was conducted on an elderly person's remains immediately after death to measure bone density in multiple sites of the same individual. We selected the skull, clavicle, lumbar vertebrae, femoral neck, and diaphysis based on the differences in bone microstructure, axial/appendicular skeletons, load/nonload-bearing bones, and ossification. A QCT-based 3D model was used to measure the volumetric BMD of selected sites in the same individual. This study is aimed at evaluating the BMD at multiple sites in the same individual and clarify the relationship between these sites. Based on the relationships identified, we aimed to examine the factors that influenced the regulatory mechanisms of bone remodeling in the elderly population.

The article "Similarities and Differences in Bone Mineral Density between Multiple Sites in the Same Individual: An Elderly Cadaveric Study" was published in 2022. Journal: Biomed Res Int.

## 2. Materials and Methods

This study was approved by the Ethics Committee of the Nagasaki University Graduate School of Biomedical Sciences (Approval No.: 15092552-2), and written informed consent was obtained from individuals (cadaver donors) and their families before death. The sample size was calculated using G∗Power version 3.1.9.2. (Universität Düsseldorf, Düsseldorf, Germany) with an effect size of 0.4, *α* = 0.05, and a power of 0.8. As a result, 44 individuals were required. Of the 89 Japanese people who died between May 2012 and December 2018, 60 that met the inclusion criteria (28 men, age: 81.6 ± 9.7 years; 32 women, age: 86.1 ± 9.5 years) were included in this study (Table 1). The exclusion criteria were as follows: (1) cases in which a good imaging limb position could not be obtained due to joint contracture; (2) cases in which bone diseases, such as bone tumors, were confirmed; and (3) cases where BMD could not be measured accurately due to trauma. All computed tomography (CT) images were read by two medical doctors, including a board-certified specialist from the Japanese Orthopaedic Association. All the experimental procedures were conducted in accordance with the principles of the Declaration of Helsinki.

### 2.1. Autopsy-Imaging Computed Tomography

All individuals were transported to the university shortly after death, and CT scans were performed to obtain skeletal data from the head to the thigh. All CT images were acquired using clinical multislice CT (Activision16, Toshiba, Tokyo, Japan; X-tube volume/current, 120 kV/100 mA; image matrix size, 512 × 512 pixels; slice thickness, 1.0 mm). In addition, a calibration phantom (B-MAS200, Kyoto Kagaku, Kyoto, Japan) containing five hydroxyapatite rods (0, 50, 100, 150, and 200 mg/cm^3^) was included in the imaging for the BMD calculation.

### 2.2. Extraction from Skeletal Target Sites and BMD Assessment

This study used MECHANICAL FINDER version 11.0 Extended Edition software (Research Center for Computational Mechanics, Tokyo, Japan) to measure BMD. This software can incorporate BMD data calculated from CT values into a 3D skeletal model built from medical Digital Imaging and Communications in Medicine data. For the 3D skeletal model, the CT value threshold was set above 300 to extract the bone contour and measure the BMD of the bone region, including the medullary cavity [18]. The BMD data that were incorporated into the 3D skeletal model were calculated using the bone density conversion equation obtained from the CT values of the calibration phantom. The included BMD data were used to calculate the average volumetric BMD (mg/cm^3^) in the bone regions within the region of interest (ROI) using functions in the software. The material data obtained using this method have previously been confirmed to be highly accurate in comparative studies with cadavers [19, 20].

The article "Similarities and Differences in Bone Mineral Density between Multiple Sites in the Same Individual: An Elderly Cadaveric Study" was published in 2022. Journal: Biomed Res Int.

From the acquired CT data, the bone ROIs (skull, clavicle, lumbar vertebra, and femur) were traced using MECHANICAL FINDER (v11.0), and a 3D bone model was constructed. A 3D model composed of 1 mm tetrahedral elements was subsequently created based on the 3D bone model.

### 2.3. BMD Assessment of the Skull

A spherical ROI with a diameter of 30 mm was placed at each measurement point to determine the BMD. The center of the sphere was set at the midpoint of the skull thickness, and the average BMD was measured. We measured the BMD at each of the defined measurement points for the frontal, temporal, and parietal bones (Figure 1). The left and right measurement points were assessed for the temporal and parietal bones, and the average value was used as the respective BMD value. The average bone density at each site was calculated and used as the skull BMD value.

### 2.4. BMD Assessment of the Clavicle, Lumbar Vertebra, and Femur

The entire left clavicle was included in the BMD measurements (Figure 2(a)). The BMD of the vertebra in the middle third of the vertebral height range was used for the lumbar vertebral measurement (Figure 2(b)). The left side of the femur was also included. The femoral neck was defined as the area between the femoral head and the lesser trochanter for the purposes of BMD measurement (Figure 2(c)). In the femoral diaphysis, the BMD was measured within a 20 mm range in the cephalocaudal direction centered on the line bisecting the adductor tuberosity and lesser trochanter (Figure 2(d)). In cases where there was a fracture of the left femoral neck (4 cases) or where accurate measurement was difficult due to artifacts caused by an implant (2 cases), the BMD of the right femur was measured.

### 2.5. Statistical Analysis

All statistical analyses were performed using the statistical software Statistical Package for the Social Sciences (version 22.0, IBM, Armonk, NY, USA). The significance level was set at *P* < 0.05. Age comparisons between men and women were performed using the unpaired *t*-test. Mean and standard deviation (SD) were used for the descriptive statistics. Two-way analysis of variance was used to determine differences according to sex and BMD at each site. Post hoc comparisons were conducted using the Bonferroni test in the event of a significant main effect. Correlation analysis was conducted using Pearson's product rate correlation coefficient and partial correlation coefficient.

The article "Similarities and Differences in Bone Mineral Density between Multiple Sites in the Same Individual: An Elderly Cadaveric Study" was published in 2022. Journal: Biomed Res Int.

## 3. Results

### 3.1. BMD Values at Each Site

The BMD measurements at each site are presented in Table 2. Two-way analysis of variance results confirmed that the variable sex had a significant effect on BMD (*P* < 0.01). Post hoc test (Bonferroni test) comparison of BMD values at each site between men and women found that the BMD values was significantly higher in men than in women at all sites (BMD values ± SD for men and women at each site, skull: 760.6 ± 131.8 vs.686.5 ± 142.0, *P* < 0.01, *F* = 7.67; clavicle: 378.2 ± 112.7 vs.304.4 ± 81.1, *P* < 0.01, *F* = 7.62; lumbar vertebra: 141.7 ± 60.0 vs.104.2 ± 38.2, *P* < 0.01, *F* = 1.97; femoral neck: 233.4 ± 82.0 vs.196.6 ± 65.4, *P* < 0.01, *F* = 1.90; and femoral diaphysis: 768.1 ± 133.8 vs.566.2 ± 191.4, *P* < 0.01, *F* = 56.92). In addition, when lumbar vertebra BMD was assessed based on the American College of Radiology and International Society for clinical densitometry diagnostic criteria for osteoporosis (BMD < 80 mg/cm^3^) [21, 22], 16.7% (*n* = 10) had osteoporosis in all individuals. By gender, 7.1% (*n* = 2) were men and 25% (*n* = 8) were women (Table 2).

### 3.2. Correlation between Age and BMD at Each Site

Table 3 shows the relationship between the BMD and age for each ROI. Correlation analysis found that BMD was negatively associated with age for all individuals in all ROIs (skull: *r* = −0.261, *P* < 0.05; clavicle: *r* = −0.490, *P* < 0.01; lumbar vertebra: *r* = −0.420, *P* < 0.01; femoral neck: *r* = −0.455, *P* < 0.01; and femoral diaphysis: *r* = −0.507, *P* < 0.01).

Table 3 and Figure 3 show the relationship between age and BMD according to sex. In men, the BMD of the lumbar vertebra and femoral neck (lumbar vertebra: *r* = −0.470, *P* < 0.05; femoral neck: *r* = −0.468, *P* < 0.05) was significantly negatively correlated with age. Conversely, in women, the clavicle, femoral neck, and femoral diaphysis were significantly negatively correlated (clavicle: *r* = −0.572, *P* < 0.01; femoral neck: *r* = −0.376, *P* < 0.01; femoral diaphysis: *r* = −0.673, *P* < 0.01) with age. In the skull, there was no significant correlation between the BMD and age in either sex (*P* > 0.05).

### 3.3. BMD Correlations at Each Site

Table 4 shows the correlation for BMD at each site in all men and women. There were significant positive correlations for all site combinations in all individuals. When the analyses were restricted to men, significant positive correlations were identified for all site combinations (femoral diaphysis and clavicle or femoral neck; both *P* < 0.05; other combinations: *P* < 0.01). No significant correlations were found between the skull and femoral neck or diaphysis in women. Significant positive correlations were found for all other combinations (lumbar vertebra and skull or clavicle; both *P* < 0.05; other combinations: *P* < 0.01).

The article "Similarities and Differences in Bone Mineral Density between Multiple Sites in the Same Individual: An Elderly Cadaveric Study" was published in 2022. Journal: Biomed Res Int.

### 3.4. Partial Correlation Analysis of BMD at Each Site

There was a moderate positive correlation between most sites. A partial correlation analysis was performed to adjust for these factors by including all measurement sites as variables and calculating the partial correlation coefficient for each site.

Table 5 shows the partial correlation of BMD at each site in all men and women. When all individuals were included, the skull was found to be significantly positively correlated with the clavicle and lumbar vertebrae (clavicle: *r* = 0.327, *P* < 0.05; lumbar vertebra: *r* = 0.295, *P* < 0.05). Additionally, significant positive correlations were found between the clavicle and femoral diaphysis (*r* = 0.354, *P* < 0.01) and between the lumbar vertebrae and femoral neck (*r* = 0.519, *P* < 0.01).

The same analysis was conducted separately for men and women, and a significant positive correlation was found between the lumbar vertebrae and femoral neck in men (*r* = 0.688, *P* < 0.01) and between the clavicle and femoral diaphysis in women (*r* = 0.559, *P* < 0.01). The skull was also positively correlated with the clavicle and lumbar vertebrae in women (clavicle: *r* = 0.484, *P* < 0.01; lumbar vertebra: *r* = 0.392, *P* < 0.05).

## 4. Discussion

Bone is a metabolically active organ that undergoes continuous remodeling throughout life. The bone remodeling cycle consists of “resorption,” in which the osteoclasts digest the old bone, and “formation,” in which the osteoblasts form a new bone until the resorbed bone is completely replaced. Bone remodeling adjusts the bone structure to meet the changing mechanical needs, repairs microdamage to the bone matrix, and prevents accumulation of the old bone. Moreover, bone remodeling plays an important role in plasma calcium homeostasis [19, 20].

Normally, bone remodeling depends on and responds to routine physiological and mechanical demands [23–25]. Physiological demand is driven primarily by endocrine fluctuations, which regulate BMD nonspecifically (systemically) in response to decreasing visceral function and nutritional interventions. Menopause-related estrogen deficiency in particular leads to decreased BMD in women [5, 26–28]. Mechanical demand is driven by habitual mechanical loading and regulates site-specific (local) BMD [29–33]. Bones that are habitually subjected to mechanical loading are more responsive to mechanical demand [34–38]. However, in elderly individuals, it is unclear whether there is any site-specificity in the regulation of age-associated bone remodeling and whether it is affected by sex.

The article "Similarities and Differences in Bone Mineral Density between Multiple Sites in the Same Individual: An Elderly Cadaveric Study" was published in 2022. Journal: Biomed Res Int.

The BMD and age were negatively correlated at all sites. Generally, BMD declines with age due to physiological factors, such as decreased kidney function, gonadal function, and mechanical factors, such as decreased activity [39–41], and our results were consistent with those of previous studies. Furthermore, we found that the correlation between BMD and age showed different site-specificity depending on sex.

We identified a significant negative correlation with age in the lumbar vertebra and femoral neck of men. Age-related bone loss has been found to be more pronounced in the trabecular bone than in cortical bone [42]. In line with these findings, we also identified a significant negative correlation with age in the lumbar vertebra and femoral neck, which are sites containing a high proportion of trabecular bones.

Conversely, in women, significant correlations between age and BMD were found in the clavicle and femoral diaphysis. Imamura et al. investigated morphological changes in the cortical bone of the femoral diaphysis with age and reported that there was no change in cortical bone thickness in men, but in women, cortical bone thickness was found to decrease with age [11]. The clavicle has a high proportion of cortical bones [43]; thus, our finding of a significant negative correlation between the BMD of the clavicle and femoral diaphysis and age in women may suggest that thinning and porosity associated with cortical bone resorption may occur in elderly women.

Notably, there was no significant correlation between skull size and age in either sex. The frontal, temporal, and parietal bones measured in this study form the calvarium, which consists of a three-layer structure in which the outer and inner plates of the cortical bone sandwich the diploë of the trabecular bone [44, 45]. The skull has a different mechanism for regulating bone remodeling than the other bones [34, 35, 45, 46]. Although the mechanism of bone remodeling regulation in the skull remains unclear, future detailed studies on the skull, which is largely unaffected by aging, may provide insights that will contribute to the treatment of osteoporosis in the future.

We found significant positive correlations between BMD sites for all combinations; however, the strength of the correlations varied by site. Additionally, partial correlation analysis, which was performed to adjust for the effects of BMD at other sites, revealed different results in men and women.

There was a significant positive correlation between the lumbar vertebrae and femoral neck in men. Because the lumbar vertebra and femur are both load-bearing bones, the regulation of bone remodeling to adapt to mechanical loading may be similar in both locations [34–38]. Additionally, the lumbar vertebra and femoral neck may undergo similar bone remodeling regulation, as they are trabecular bone-rich regions with similar microstructures.

The article "Similarities and Differences in Bone Mineral Density between Multiple Sites in the Same Individual: An Elderly Cadaveric Study" was published in 2022. Journal: Biomed Res Int.

Alternatively, in women, we identified a positive correlation between the clavicle and femur diaphysis and BMD. Both the clavicle and femoral diaphysis contain a high proportion of cortical bones and have similar microstructures. This finding is unique to women and can be attributed to the fact that women in our study were at least 10 years postmenopausal. Bone mass in women's trabecular bone declines rapidly immediately after menopause, and then the pace of decline slows [39, 47]. It is possible that the women in this study were already in the slow period of trabecular bone loss, and the results may indicate that thinning and porosity associated with cortical bone loss may be progressive in elderly women. Furthermore, there was a significant correlation between the clavicle, a nonweight-bearing bone, and the femoral diaphysis, a weight-bearing bone, suggesting that morphological changes with cortical bone loss may be progressive, regardless of whether the bone is weight-bearing or non-weight-bearing. However, because this study did not include individuals before and after menopause, it was not possible to further clarify changes in the regulation of trabecular and cortical bone remodeling in women. Future studies over a wide range of ages may reveal changes in the regulation of bone remodeling between trabecular and cortical bone in women.

Furthermore, a significant positive correlation between the BMDs of the skull and clavicle was identified in women. The skull and clavicle are both nonweight-bearing bones and thus may be affected by similar regulation of bone remodeling. Moreover, since the area where the BMD of the skull was measured in this study was relatively rich in cortical bone [44], it is possible that the correlation with the clavicle was due to the similarity of the bone microstructure. Additionally, both the skull and part of the clavicle are classified as intramembranous ossification [48, 49], which means that the ossification process may affect bone remodeling regulation. However, since the sites where the BMD of the clavicle was measured in this study included endochondral ossification sites, future investigations of BMD in different parts of the clavicle will help clarify the effects of different ossification processes on bone remodeling regulation.

The article "Similarities and Differences in Bone Mineral Density between Multiple Sites in the Same Individual: An Elderly Cadaveric Study" was published in 2022. Journal: Biomed Res Int.

Our study had some limitations, because we only had access to information on age at death, sex, and cause of death for the cadavers included in this study, we could not consider the influence of medical history, lifestyle history, and medication. Therefore, the BMD measured in this study may have been affected by BMD-modifying diseases, such as hyperparathyroidism or diabetes, or drugs, such as bisphosphonates. This point may be further elucidated by testing bone metabolism markers and cell histological data. Further, since the BMD measurement method used in this study is different from the QCT used in clinical practice, the measurements cannot be compared between studies. However, this is not a problem because this study is aimed at investigating the correlation of BMD between sites and did not compare the absolute values of the measurements with those of other studies. Additionally, because this study was an analysis of cadavers immediately after death, the samples were biased toward the elderly, and comparisons before and after menopause were not possible. However, the results of the National Center for Health Statistics (U.S.) study of the prevalence of osteoporosis in adults aged 65 and over (the prevalence of osteoporosis: 17.7% for total, 5.7% for men, and 27.1% for women) [50] and the results of the prevalence of osteoporosis in the current study subjects are similar; these study samples may be representative of the general geriatric population.

Unless clinically necessary, it is difficult to obtain whole-body BMD data using CT images due to radiation exposure and other problems. In this regard, our study provides valuable basic data as it investigates the relationship between BMD at multiple sites from the head to the thigh in the same person by using CT images taken over a wide area immediately after death. The effects of various factors on the regulation of bone remodeling at each site identified in this study will contribute to the elucidation of the pathological mechanisms of fragility fractures in the elderly population. Our results suggest the necessity of cortical bone assessment as well as trabecular bone assessment for BMD measurement in elderly women. BMD assessment using a 3D model with QCT in this study is expected to collect a large amount of data on BMD if generalized because BMD assessment of body parts can be easily performed from medical CT images.

## 5. Conclusions

The correlation between age and BMD suggests the possibility of progressive trabecular bone loss in elderly men and progressive cortical bone loss in elderly women. The correlations of BMD among the different sites suggest that the effect of bone remodeling regulation may differ depending on whether the bone is (1) load bearing or nonload bearing, (2) trabecular or cortical, and (3) intramembranous or endochondral ossification. The similarities and differences in site-specific bone remodeling regulation identified in this study may help elucidate the pathological mechanisms of osteoporosis and lead to the development of preventive and therapeutic measures. Additionally, the sex differences in bone remodeling regulation identified in this study indicate the importance of cortical bone assessment in BMD testing, particularly in elderly women.

The article "Similarities and Differences in Bone Mineral Density between Multiple Sites in the Same Individual: An Elderly Cadaveric Study" was published in 2022. Journal: Biomed Res Int.

## Figures and Tables

**Figure 1:** Schema of the bone mineral density (BMD) measurement points. The lower panel shows the actual regions of interest. The center of a sphere of 15 mm radius was aligned with the center of bone thickness at the measurement point, and the average BMD (mg/cm^3^) of the bone contained in the sphere was used as the BMD. (a) BMD measurement of the frontal bone, where the midpoints of Bregma and Nasion were defined as the measurement points (red dots). (b) BMD measurement of the temporal and parietal bones. Measurement point was defined as the midpoint of porion and (iii) for the temporal bone and the intersection of the superior temporal line and (ii) for the parietal bone (red dots). (i) Frankfurt plane, (ii) plane orthogonal to the Frankfurt plane and passing through the Porion, and (iii) point of intersection of (ii) and the scaly suture.

**Figure 2:** The sites of bone mineral density (BMD) measurement for the clavicle, lumbar vertebra, femoral neck, and femoral diaphysis. (a) In the clavicle, the region of interest (ROI) was set at the left side of the clavicle; (b) in the lumbar vertebra, the ROI was set at the middle one-third of the height of the vertebral body at L2; (c) in the femoral neck, the ROI was set at the area between the femoral head and lesser trochanter; (d) in the femoral diaphysis, the ROI was set at 20 mm in the cephalocaudal direction centered on the line bisecting from the lesser trochanter to the adductor tuberosity.

**Figure 3:** Scatter plots showing the relationship between age and bone mineral density (BMD) by sex. The blue dots represent men, and the orange dots represent women. The dotted line indicates a linear regression.

**Table 1:** Sex and the generational distribution of individuals.

	Men	Women
60–69	4	2
70–79	7	4
80–89	12	13
90–99	5	13
Total	28	32
Average age	81.6 ± 9.7	86.1 ± 9.5

There were no significant differences in age between men and women.

**Table 2:** Bone mineral density (BMD) values for each site and prevalence of osteoporosis.

	All individuals (*n* = 60)	Men (*n* = 28)		Women (*n* = 32)
Skull (mg/cm^3^)	721.1 ± 141.2	760.6 ± 131.8	>^∗∗^	686.5 ± 142.0
Clavicle (mg/cm^3^)	338.9 ± 103.2	378.2 ± 112.7	>^∗∗^	304.4 ± 81.1
Lumbar vertebra (mg/cm^3^)	121.7 ± 52.6	141.7 ± 60.0	>^∗∗^	104.2 ± 38.2
Femoral neck (mg/cm^3^)	213.8 ± 75.3	233.4 ± 82.0	>^∗∗^	196.6 ± 65.4
Femoral diaphysis (mg/cm^3^)	660.4 ± 194.3	768.1 ± 133.8	>^∗∗^	566.2 ± 191.4
Osteoporosis (%)	16.7 (*n* = 10)	7.1 (*n* = 2)		25 (*n* = 8)

The diagnosis of osteoporosis was determined from BMD of the lumbar spine based on the diagnostic criteria of the American College of Radiology and International Society for clinical densitometry (BMD < 80 mg/cm^3^). The BMD values for each site were analyzed with a two-way (sites × sex; 5 × 2) analysis of variance with repeated measures. In the event of a significant main effect, post hoc comparisons were conducted using the Bonferroni test. ^∗∗^*P* < 0.01.

The article "Similarities and Differences in Bone Mineral Density between Multiple Sites in the Same Individual: An Elderly Cadaveric Study" was published in 2022. Journal: Biomed Res Int.

**Table 3:** Relationship between bone marrow density (BMD) of each site and age.

	*r* value		
	All individuals (*n* = 60)	Men (*n* = 28)	Women (*n* = 32)
Skull	−0.261^∗^	n.s.	n.s.
Clavicle	−0.490^∗∗^	n.s.	−0.572^∗∗^
Lumbar vertebra	−0.420^∗∗^	−0.470^∗^	n.s.
Femoral neck	−0.455^∗∗^	−0.468^∗^	−0.376^∗^
Femoral diaphysis	−0.507^∗∗^	n.s.	−0.673^∗∗^

The numbers indicate Pearson's product rate correlation coefficient. ^∗^*P* < 0.05 and^∗∗^*P* < 0.01; n.s.: not significant.

**Table 4:** Correlation coefficients of bone mineral density (BMD) from different sites.

	Skull	Clavicle	Lumbar vertebra	Femoral neck
All individuals				
Clavicle	0.555^∗∗^			
Lumbar vertebra	0.550^∗∗^	0.621^∗∗^		
Femoral neck	0.425^∗∗^	0.601^∗∗^	0.730^∗∗^	
Femoral diaphysis	0.359^∗∗^	0.606^∗∗^	0.560^∗∗^	0.543^∗∗^
Men				
Clavicle	0.576^∗∗^			
Lumbar vertebra	0.601^∗∗^	0.637^∗∗^		
Femoral neck	0.549^∗∗^	0.549^∗∗^	0.827^∗∗^	
Femoral diaphysis	0.492^∗∗^	0.417^∗∗^	0.540^∗∗^	0.455^∗^
Women				
Clavicle	0.461^∗∗^			
Lumbar vertebra	0.423^∗∗^	0.428^∗∗^		
Femoral neck	n.s.	0.594^∗∗^	0.518^∗∗^	
Femoral diaphysis	n.s.	0.674^∗∗^	0.474^∗∗^	0.575^∗∗^

The numbers indicate Pearson's product rate correlation coefficient. ^∗^*P* < 0.05 and^∗∗^*P* < 0.01; n.s.: not significant.

**Table 5:** Partial correlation coefficients calculated from the bone mineral density (BMD) of each site.

	Skull	Clavicle	Lumbar vertebra	Femoral neck
All individuals				
Clavicle	0.327^∗^			
Lumbar vertebra	0.295^∗^	n.s.		
Femoral neck	n.s.	n.s.	0.519^∗∗^	
Femoral diaphysis	n.s.	0.354^∗∗^	n.s.	n.s.
Men				
Clavicle	n.s.			
Lumbar vertebra	n.s.	n.s.		
Femoral neck	n.s.	n.s.	0.688^∗∗^	
Femoral diaphysis	n.s.	n.s.	n.s.	n.s.
Women				
Clavicle	0.484^∗∗^			
Lumbar vertebra	0.392^∗^	n.s.		
Femoral neck	n.s.	n.s.	n.s.	
Femoral diaphysis	n.s.	0.559^∗∗^	n.s.	n.s.

The numbers indicate partial correlation coefficient. ^∗^*P* < 0.05 and ^∗∗^*P* < 0.01; n.s.: not significant.A.

The article "Similarities and Differences in Bone Mineral Density between Multiple Sites in the Same Individual: An Elderly Cadaveric Study" was published in 2022. Journal: Biomed Res Int.

## Data Availability

The material data used to support the findings of this study are restricted by the Nagasaki University Graduate School of Biomedical Sciences in order to protect participants' privacy. Data are available from Keita Nishi (k-nishi@nagasaki-u.ac.jp) for researchers who meet the criteria for access to confidential data.
